RETRACTED

# Location and Effect of Bone Cement in Percutaneous Vertebroplasty for Osteoporotic Vertebral Compression Fractures

**DOI:** 10.1155/2022/6127620

**Published:** 2022-06-26

**Authors:** Xu Ding, Qianfa Zhang, Yi Zhao, Jian Wang

**Affiliations:** Department of Orthopedic Surgery, Zhongshan Hospital Wusong Branch, Fudan University, Shanghai 200940, China

## Abstract

In this study, the effectiveness and use of bone cement are thoroughly elaborated, and the role of bone cement on percutaneous vertebroplasty (PVP) fixed joints and its distribution on PVP are also elucidated. The aim of this study was to investigate the effect of unilateral and bilateral bone cement distribution on the clinical efficacy of PVP in the treatment of osteoporotic vertebral compression fractures (OVCF) of the thoracolumbar spine. A total of 60 patients with thoracolumbar OVCF (T11-L2) hospitalized in our hospital from January 2020 to January 2021 were studied. All patients had thoracolumbar OVCF. Under the guidance of the C-arm machine, unilateral PVP was performed. According to the distribution of bone cement across the midline, the patients were divided into two groups: the unilateral group (37 cases): bone cement was distributed on one side of the midline of the vertebral body, and the bilateral group (23 cases): bone cement was distributed on both sides of the midline. Visual analogue scale (VAS), vertebral height recovery values, and preoperative and postoperative Cobb's angle were recorded at 3 days, 1 month, 3 months, and 6 months. The differences between the two groups were compared and analyzed to evaluate the clinical efficacy. There was a statistically significant difference in VAS scores between the two groups before and after surgery (*P* < 0.05), but there was no statistically significant difference in VAS scores between the two groups at 3 days, 1 month, 3 months, and 6 months after surgery (*P* > 0.05). There were statistically significant differences in vertebral height recovery value and Cobb's angle between the two groups before and after surgery (*P* < 0.05).

## 1. Introduction

PVP was first successfully applied clinically in 1984 by French doctors Deramand and Galibert [1] to treat bone damage occurring in the cervical vertebrae. At that time, it was not used for vertebral fractures but lesions caused by hemangioma. In 1993, American doctors first used PVP to treat OVCF under this premise and obtained the same efficacy. Since then, PVP has been widely promoted and applied at home and abroad for its advantages of early effective pain relief, avoidance of complications caused by long-term bed rest, and small trauma. With the rapid development of the social economy and the continuous improvement of human living standards, society is gradually aging, and China has also entered a high incidence of osteoporosis. The incidence of osteoporosis in people over 60 years old is about 56%. Among the complications of osteoporosis, the most common is vertebral compression fracture [2], namely, OVCF, whose main clinical manifestations are severe pain in the affected area and dysfunction of functional activities. According to statistics [3], patients with inconspicuous symptoms account for about 2/3 of clinical patients, while patients with obvious symptoms account for about 1/3. Therefore, it is the treatment required for this disease to actively relieve the pain symptoms of patients, restore their self-care ability as soon as possible, and improve their activity function.

RETRACTED

Literature has shown that PVP can significantly relieve lumbar and back pain symptoms. The second day after the operation can be used to get out of the ground to reduce the difficulty of nursing and achieve rapid recovery [4–6]. However, it has been found clinically that there are still some patients with low back pain after PVP who have recurrent symptoms and even cannot be relieved, and the factors affecting the clinical efficacy are not clear at present [7–9]. Therefore, the focus of this study was to observe the effect of the unilateral or bilateral distribution of bone cement on the clinical efficacy after PVP. In a retrospective study, 60 patients with OVCF treated by PVP in our hospital from January 2020 to January 2021 were divided into a unilateral group and bilateral group according to the unilateral or bilateral distribution of bone cement, and the relevant indicators of the two groups were compared to explore the clinical efficacy.

## 2. Methods

### 2.1. Participants

Sixty patients with thoracolumbar (T11-L2) OVCF hospitalized in our hospital from January 2020 to January 2021 were collected to gather the experimental values.

(i) Inclusion criteria
  1. Met the diagnostic criteria of osteoporosis
  2. Have a clear history of trauma and inducement
  3. Acute injury (patient from injury to surgical within 2 weeks)
  4. The vertebral segment of the disease was consistent with the clinical symptoms and physical examination and the clinical presentation consistent with radiographic cues, and all were thoracolumbar single vertebral fractures
  5. Magnetic resonance imaging (MRI) examination confirmed fresh vertebral fracture when necessary
(ii) Exclusion criteria
  1. Multilevel thoracolumbar compression fracture
  2. Vertebral compression fracture caused by tumor
  3. Those who take hormones for a long time
  4. Postoperative bone cement leakage occurred in the intervertebral disc
  5. Previous vertebral augmentation and other spinal surgeries
  6. Patients with coagulation abnormalities, poor cardiopulmonary function, and poor tolerance

RETRACTED

### 2.2. Surgical Method

After disinfecting the skin and local anesthesia, the needle tip is inserted on the pedicle side of the spine, and a small incision of about 0.5 cm is inserted into the pedicle root of the unlabeled side; the needle is penetrated from the pedicle into the center of the vertebral body. (conventional puncture method: the puncture point is located at the outer upper edge of the projection of the pedicle in orthostatic perspective). From a lateral perspective, the needle continues to enter the anterior 1/3 position of the vertebral body in the direction of the pedicle. The bone cement was adjusted, and about 4~5 mL of bone cement was injected into each vertebral body. Orthogonal fluoroscopy shows a well-distributed vertebral cement to completely cover the wound.

## 3. Observed Indicator

The following indexes were observed: VAS score, vertebral height recovery value, and Cobb's angle on the sagittal plane of the affected vertebra (Cobb's angle from the upper-end plate of the affected vertebra to the lower endplate of the affected vertebra) before and after surgery at 3 d and 1, 3, and 6 months. The formula of the recovery rate of anterior vertebral height was [(Ha/Hp) postoperative − (Ha/Hp) preoperative] × 100%. The recovery rate of central vertebral height was calculated as follows: [(Hm/Hp) postoperative − (Hm/Hp) preoperative] × 100%. This study considered no improvement as vertebral height recovery of less than 3%. (Ha: height of anterior margin of a vertebral body; Hm: height of middle margin of a vertebral body; and Hp: height adjacent to posterior margin of the vertebral body).

### 3.1. Statistical Analysis

SPSS17.0 statistical software package was used for statistical analysis. Measurement data were expressed as mean ± standard deviation (*X* ± *S*); a comparison was performed by *T*-test; *P* < 0.05 was considered statistically significant.

## 4. Results

### 4.1. General Information Comparison

A total of 60 patients were included, including 21 males and 39 females. Their ages ranged from 56 to 82 years, with an average of 72.57 years. The disease course ranged from 1 to 12 days, with an average of 3.68 days. There were 37 cases in the unilateral group, including 11 males and 26 females, with an average age of 73.8 ± 2.7 years. There were 6 cases of T11 vertebral body, 17 cases of T12 vertebral body, 12 cases of lumbar 1 vertebral body, and 2 cases of lumbar 2 vertebral body. In the bilateral group, there were 23 patients: 7 males and 16 females, with an average age of 73.6 ± 3.6 years, 3 T11 vertebrae, 10 T12 vertebrae, 9 lumbar, 1 vertebrae, and 1 lumbar 2 vertebrae. Both groups had no symptoms and signs of spinal nerve compression before surgery. X-ray showed wedge-shaped changes, CT showed a complete posterior wall of a vertebral body, and an MRI showed a low signal in T1W1 and a high signal in T2W1 of an affected vertebral body. There was no significant difference in age and gender between the two groups (*P* > 0.05), indicating comparability.

RETRACTED

### 4.2. Comparison of VAS Scores

There was a statistically significant difference in VAS scores between the two groups before and after surgery (*P* < 0.05), but there was no statistically significant difference in VAS scores between the two groups before, 3 days after surgery, 1 month after surgery, 3 months after surgery, and 6 months after surgery (*P* > 0.05) (see Table 1).

### 4.3. Comparison with Preoperative

#### 4.3.1. Vertebral Height Recovery Value (MM) Score Comparison

There was a statistically significant difference in vertebral height recovery value between the two groups before and after surgery (*P* < 0.05), and there was a statistically significant difference in vertebral height recovery value between the two groups (*P* < 0.05) (see Table 2).

### 4.4. Cobb's Angle (°) Score Comparison

There was a statistically significant difference in Cobb's angle between the two groups before and after the operation (*P* < 0.05), but there was no statistically significant difference in Cobb's angle between the two groups (*P* > 0.05) (see Table 3).

### 4.5. Discussion

The degree of osteoporosis, the viscosity of bone cement, injection pressure, fracture degree, angle, and depth of puncture needle are considered to be the main influencing factors of bone cement distribution [9, 10]. Studies of PVP from unilateral and bilateral pedicles [11, 12] have been found to have similar long-term clinical effects, but this study concluded that the primary purpose of treating compressive vertebral fractures was to relieve pain and restore vertebral height and adjacent vertebral fractures. Whether PVP surgery or not, the pain relief can be relieved in the long term, but the recovery of vertebral height is difficult. Matsuura et al. [13] believe that unilateral PVP can take advantage of the short operation time, less radiation, and less trauma. However, unilateral bone cement entry causes an uneven distribution in the vertebral body, making the bone cement unable to fill the fracture line fully. Therefore, this study suggests that bilateral bone cement filling should be ensured as much as possible in PVP surgery [14–16]. When bone cement is evenly distributed bilaterally in the vertebral body, there is no significant difference in clinical efficacy between unilateral and bilateral punctures. Li et al. [17] and Wei et al. [18] also have the same view.

RETRACTED

In this study, patients with thoracolumbar fractures with similar clinical characteristics were enrolled and divided into unilateral and bilateral groups based on the distribution of bone cement on one or both sides of the vertebral body. There were statistically significant differences in VAS scores between each group before and after surgery (*P* < 0.05), but there were no statistically significant differences between groups before, 3 days after surgery, 1 month after surgery, 3 months after surgery, and 6 months after surgery (*P* > 0.05). The results showed that the postoperative VAS scores of bone cement distribution on one side of the vertebral body and bone cement distribution on both sides of the vertebral body were significantly improved compared with preoperative, achieving the effect of bone analgesia. In the middle and late follow-up, the bone cement distribution did not affect the VAS score. There were statistically significant differences in vertebral height recovery value and Cobb's angle between the unilateral group and the bilateral group before and after surgery (*P* < 0.05), and there were statistically significant differences in vertebral height recovery value and Cobb's angle between the bilateral group and the unilateral group before and after surgery (*P* < 0.05), indicating that the degree of compressed vertebral deformity could be improved in both the unilateral group and the bilateral group after surgery. The comparison of postoperative vertebral height recovery values between the unilateral group and bilateral group was statistically significant (*P* < 0.05), indicating that bilateral distribution of bone cement has a better effect on the recovery and maintenance of vertebral height.

In summary, the vertebral height recovery value and Cobb angle remain stable during the simultaneous placement. In patients with OVCF, the bilateral bone cement distribution has a good effect on preventing further collapse and fracture of adjacent vertebral bodies within the second half of the year after PVP. It has certain clinical significance for maintaining vertebral stability. However, the bilateral distribution of the unilateral approach to complete the cement requires a large abduction puncture angle, which can easily lead to damage to the inner wall and nerves of the pedicle and leakage of bone cement. Although the bilateral approach takes a long time and has a lot of radiation and great trauma, it only needs a small abduction angle to achieve bilateral distribution of bone cement, thus reducing the risk of nerve injury and bone cement leakage. In clinical PVP, unilateral or bilateral puncture has advantages and disadvantages, which should be determined according to the specific condition and the status of the responsible vertebral body. However, the bilateral distribution of bone cement certainly has a certain clinical significance on vertebral recovery height and Cobb's angle.

RETRACTED

## 5. Conclusion

Whether the bone cement is distributed in the midline, PVP can achieve an effective clinical effect. However, the clinical effect of bone cement distributed on both sides of the midline of the vertebral body is better than that of bone cement distributed on the midline side of the vertebral body.

## Figures and Tables

**Table 1:** Comparison of preoperative and postoperative VAS scores between two groups (*X* ± *S*).

Group	*N*	Before surgery	3 days after surgery	1 month after surgery	3 months after surgery	6 months after surgery
Unilateral group	37	7.63 ± 0.75	3.76 ± 0.68^∗^	2.58 ± 0.48^∗∗^	2.20 ± 0.45^∗∗^	2.06 ± 0.39^∗∗^
Bilateral group	23	7.68 ± 0.77	3.52 ± 0.57^∗^	2.44 ± 0.43^∗∗^	2.24 ± 0.57^∗∗^	2.14 ± 0.52^∗∗^

^∗^ *P* < 0.05; comparison between groups: ^∗∗^*P* > 0.05.

**Table 2:** Comparison of preoperative and postoperative vertebral height recovery (mm) scores between the two groups (*X* ± *S*).

Group	Index	Before surgery	3 days after surgery	1 month after surgery	3 months after surgery	6 months after surgery
Unilateral group	Leading edge of the central	17.6 ± 5.0	19.3 ± 4.7^∗^	19.2 ± 3.9^∗∗^	19.1 ± 4.2^∗∗^	19.1 ± 4.0^∗∗^
		12.5 ± 4.1	14.5 ± 4.3^∗^	14.3 ± 4.1^∗∗^	14.2 ± 4.0^∗∗^	14.2 ± 3.9^∗∗^
Bilateral group	Leading edge of the central	17.5 ± 5.3	20.6 ± 5.4^∗^	20.5 ± 5.2^∗∗^	20.4 ± 5.0^∗∗^	20.4 ± 5.0^∗∗^
		12.3 ± 3.9	15.5 ± 4.4^∗^	15.4 ± 4.3^∗∗^	15.4 ± 4.1^∗∗^	15.4 ± 4.1^∗∗^

**Table 3:** Comparison of Cobb's angle (°) scores between the two groups before and after the operation (*x* ± *s*).

Group	*N*	Before surgery	3 days after surgery
Unilateral group	37	22.68 ± 5.06	21.44 ± 3.27
Bilateral group	23	23.42 ± 3.21	21.08 ± 2.99

## Data Availability

The datasets used and analyzed during the current study are available from the corresponding author upon reasonable request.
